The article "Investigation of Artery Wall Elasticity Effect on the Prediction of Atherosclerosis by Hemodynamic Factors" was published in 2022. Journal: Appl Bionics Biomech.

# Investigation of Artery Wall Elasticity Effect on the Prediction of Atherosclerosis by Hemodynamic Factors

**DOI:** 10.1155/2022/3446166

**Published:** 2022-04-05

**Authors:** Rasool Kalbasi, Bahador Sharifzadeh, Mehdi Jahangiri

**Affiliations:** ^1^Department of Mechanical Engineering, Najafabad Branch, Islamic Azad University, Najafabad, Iran; ^2^Department of Mechanical Engineering, Shahrekord Branch, Islamic Azad University, Shahrekord, Iran

## Abstract

Atherosclerosis is a vascular disease in which some parts of the artery undergo stenosis due to the aggregation of fat. The causes and location of stenosis can be determined using fluid mechanics and parameters such as pressure, effective wall shear stress, and oscillatory shear index (OSI). The present study, for the first time, numerically investigates the pulsatile blood flow inside arteries with elastic and rigid walls in simple and double stenosis (80% stenosis) by using *k*-*ω* model and physiological pulse. The reason for applying the *k*-*ω* model in the present study was to provide more consistent results with clinical results to improve the accuracy in estimating atherosclerosis disease. The investigation of the time-mean wall shear stress indicated that for double stenosis, the difference between the results of the rigid and elastic artery assumptions is greater than the case of simple stenosis, so that this difference percent can be up to 2.5 times. In addition, the results showed that the pressure drop for the first stenosis is greater than the second stenosis, by 810 Pa (for solid artery) and 540 Pa (for elastic artery). The results also revealed that for simple stenosis, the length of the diseases prone zone in the elastic artery is 21% longer than the rigid one which this figure for double stenosis is calculated to be about 40%. Comparing the results of the simple stenosis with double, one affirmed that the artery wall thickness growth for case of double stenosis is greater than that of the single one.

## 1. Introduction

Atherosclerosis is one of the most common vascular diseases in which fat aggregates in some parts on the artery wall and decreases the cross-section. In this case, the artery is said to have stenosis. The stenosis inside the artery creates a path with a high hydrodynamic resistance, which leads to a lower blood flow rate. On the other hand, the stenosis inside the artery makes the blood flow turbulent. Therefore, the deposition rate rises, leading to a higher disease growth rate. The formation points, procedure, and schedule of occlusion are dependent on hemodynamic parameters. Fluid mechanics can be employed to obtain hemodynamic parameters. With the help of parameters such as pressure, effective wall shear stress, and oscillatory shear index (OSI), the causes and locations of stenosis in the artery can be found [1]. Many studies simulated the artery blood flow inside a rigid wall. Chul and Ryou [2] modeled the unsteady, non-Newtonian, and turbulent blood flow in a bifurcated artery with 75% stenosis by using the modified *k*-*ε* model. They assumed a rigid wall. They investigated the effect of the body's periodic acceleration on the turbulence and wall shear stress (WSS). The results demonstrated that the body's periodic acceleration increased turbulence, thereby changing the volumetric flow rate and blood velocity. WSS was also dependent on the periodic acceleration and followed an incremental trend. Li et al. [3] simulated the Newtonian and compressible blood flow in an artery with a rigid wall by computational fluid mechanics (CFD). They assumed a very high stenosis degree and a bifurcated artery. They provided results for Reynolds numbers from 200 to 900. It was observed that the peak mean-time WSS was 73 Pa. According to the contours, the regional stenosis throat had a high WSS. Hye and Paul [4] investigated the incompressible, Newtonian, turbulent, and steady flow inside a rigid-walled artery with 75% stenosis. They also investigated the effects of rotational and nonrotational flows. They used the *k*-*ω* model.

The article "Investigation of Artery Wall Elasticity Effect on the Prediction of Atherosclerosis by Hemodynamic Factors" was published in 2022. Journal: Appl Bionics Biomech.

Tabe et al. [5] focused on the process of a laminar flow becoming a turbulent flow, assuming a Newtonian and incompressible flow. They used arteries with 50% and 75% simple stenosis. They used the *k*-*ω* SST model for turbulent regions. They used the section-to-section simulation method and showed that this method could satisfactorily predict the behavior of an artery with stenosis.

The radius of an elastic-walled artery can change, and an increase or decrease in the flow cross-section considerably influences the WSS. The artery change range is 5-7% among old people and 8-11% among young people. A change in the artery cross-section can cause a compressive wave inside the artery, whose effect can reach to the downstream of the flow. The cardiovascular system is the best fluid-solid interaction example in nature. Ahmed and Giddens [6] experimentally studied an oscillating speed field blocked by axially symmetric stenosis. They showed that there was no permanent flow separation poststenotic region even for the largest stenosis, compared to a steady flow. The results demonstrated that the WSS values were larger near the throat than in the poststenotic region. Turbulence happened only for the 75% stenosis case. Pielhop et al. [7] experimentally investigated the presence of symmetric simple congestion on the flow field. Experimental observations show that the parameters after clogging are very different from those before. Sadeghi et al. [8] proposed a new empirical method by which stenosis-caused gradients and compressive waves can be obtained.

The article "Investigation of Artery Wall Elasticity Effect on the Prediction of Atherosclerosis by Hemodynamic Factors" was published in 2022. Journal: Appl Bionics Biomech.

Jahangiri et al. [9] numerically investigated the hemodynamic parameters of the pulse blood flow in an artery with 80% stenosis. They investigated four cases, based on turbulent and laminar flows and rigid and elastic walls. The turbulent flow was simulated using the *k*-*ε* and *k*-*ε* RNG models. The contours showed that the maximum circumferential stress occurred in the prestenosis region, and the minimum circumferential stress happened in the throat. The difference between the elastic and rigid walls was small for the laminar flow. However, it became larger when the flow became turbulent.

In another study, Jahangiri et al. [10] investigated a laminar/turbulent pulse blood flow inside an elastic-walled artery with stenosis. They mainly focused on the effect of wall elasticity/rigidity on the laminar and turbulent flows. The turbulent blood flow was simulated using the *k*-*ε* Standard and *k*-*ε* RNG models. The *k*-*ε* Standard model showed better empirical consistency. According to the observations and calculations, a laminar flow assumption is realistic to up to 70% stenosis. However, for stenosis more than 80%, turbulent methods should be used to simulate the flow field.

Sharifzadeh et al. [11] investigated the effects of using turbulence models (*k*-*ε* and *k*-*ω*) on blood flow inside a rigid wall artery with simple and double stenosis. They used finite volume method for simulation and studied the variations of oscillatory shear index (OSI) and mean wall shear stress (mean WSS) as well as reverse flow region length. Their results revealed that probability of arterial wall collapse (due to negative pressure) in *k*-*ω* approaches is higher than *k*-*ε* method. They also found that *k*-*ε* model estimated a higher plaque growth rate than the *k*-*ω* one.

Moradicheghamahi et al. [12] investigated the turbulent flow through the carotid bifurcation and used the *k*-*ε* and *k*-*ω* turbulence models. Their results showed that the effects of the rigid/elastic artery wall is more important than the Newtonian/non-Newtonian behavior of the blood. In addition, the Newtonian/non-Newtonian behavior of blood has a greater effect than the laminar/turbulent blood flow.

Freidoonimehr et al. [13] examined blood flow through a rigid coronary artery with asymmetric stenosis using physiological pulses. The effects of stenosis geometry, pulsed inlet flow, and turbulence caused by blood flow through stenosis were examined. Their results affirmed that a new stenosis was likely to form at 10D downstream the previous stenosis.

The article "Investigation of Artery Wall Elasticity Effect on the Prediction of Atherosclerosis by Hemodynamic Factors" was published in 2022. Journal: Appl Bionics Biomech.

Abdelwahab et al. [14] described a mathematical and numerical model for blood solidification and its rupture in a diseased artery in order to the comparison between stenosis and aneurysm segments through the artery. They formulated the interaction between the blood flow and wall of artery was. The blood flow is considered as a micropolar incompressible fluid with heat and mass transfer under the control of electro-osmotic and electromagnetic forces through an artery which contains stenosis and aneurysms. They illustrated that as a result of exist the stenosis and aneurysm regions, the flow rate higher in aneurysm than stenosis and so the resistance and wall shear stress are be less in aneurysm than stenosis.

Ramadan et al. [15] investigated the impacts of heat transfer and electroosmotic force on Phan-Thien–Tanner fluid, including gold nanoparticles. The Phan-Thien–Tanner fluid model was utilized to examine the rheology of blood moving through a tapered artery along with stenosis. The flow was considered to be incompressible and irrotational. They observed that a great change in the gold nanoparticle concentration after enhancing the Joule heating parameter, because the gold nanoparticles absorb the internal heat and lean to propagate in the converse stream.

Elogail and Mekheimer [16] developed a new mathematical model simulating microvascular blood flow with oxygen-repellent microorganisms and nanoparticles in the presence of heat and mass transfer coupled with progressive patterns of microorganisms. In this study, the blood viscosity was considered to vary with temperature, nanoparticle concentration, and shear strain. They found that increasing in oxygen concentrations causes the microorganism density to increase in the direction towards the hypoxic tumor regions; even a reduction in blood viscosity is regarded.

In the previous studies, the researchers demonstrated that the turbulence *k*-*ε* model cannot simulate the reverse flow and predict the exact location of the disease as well as the *k*-*ω* model. The present study compares the turbulence *k*-*ω* model for rigid and elastic walls. Furthermore, the elastic and rigid wall assumptions were not investigated for double stenosis. Hence, it is investigated in this study. This study is mainly focused on the importance of the turbulence model type and artery wall model type. Finally, it will be found whether the turbulence model is more important or the rigidity/elasticity of the artery wall.

The present work is in the development of the previous works of Jahangiri et al. [9, 10]. Also, the pressure pulse used as the output boundary condition in the present work is derived from the experimental results. In addition, to justify the results of the present work, the clinical results of others have been used, and they have been used to predict the development and development of atherosclerosis. Therefore, the results of the present numerical work are very valuable and can help the surgeons and researchers in this field. This method can be used to answer the question of whether surgery is needed for the patient or not or where are the critical sites of the disease and how does the disease spread and develop.

The article "Investigation of Artery Wall Elasticity Effect on the Prediction of Atherosclerosis by Hemodynamic Factors" was published in 2022. Journal: Appl Bionics Biomech.

## 2. Problem Description

The present study investigates the blood flow inside an artery with a rigid/elastic wall. In order to bring the results of the present work more in line with the experimental ones and also to bring the predictions of the present work closer to the clinical conditions, the physiological pressure pulse obtained from the experimental work has been used. Therefore, the geometry of the present work is also consistent with the experimental one. Also, producing real elastic artery is a very difficult process due to the available facilities.

In the artery, there is one (Figure 1(a)) or two (Figure 1(b)) stenosis. The research has shown that the flow will be turbulent at stenosis larger than 80% [9]. The present study chooses 80% of stenosis to have turbulent flow. The artery equation in the stenosis zone is shown as [17]:

(1) $$\begin{array}{c} \frac{R\left(z\right)}{R_{0}}=1-\left(\frac{R_{0}-R_{0,t}}{2R_{0}}\right)\times \left(1+\cos\frac{2\pi \left(z-z_{m}\right)}{L_{st}}\right). \end{array}$$

The blood viscosity and density were considered as 0.0033 Pa.s and 1050 kg/m^3^, respectively. Furthermore, because the wall is elastic in a part of the calculations, it is necessary to know its displacement. The Poisson's ratio, density, elasticity modulus, and thickness of the artery are considered as 0.49, 1300 km/m^3^, 910 kPa, and 0.0005 m, respectively [18].

In the present work, using physiological pulses, the velocity and pressure (derived from laboratory tests) were defined as input and output boundary conditions, respectively, and then, hemodynamic parameters were investigated. To analyze the results and predict the development or spread of the disease, the clinical results of other researchers were used to validate and compare the results. Therefore, analyzing the results of the present work by using the clinical results of other researchers as well as using physiological pulses can be considered innovations.

## 3. Governing Equations

It is important to obtain the velocity field (vertical and horizontal velocity components) to estimate the shear stress on the artery wall, because shear stress between the artery wall and the blood flow is caused by the velocity difference. The velocity field is obtained from the balance between the forces applied to each molecule and its momentum variations. The momentum equation is the balance between applied forces (left-hand side) and changes in momentum (right-hand side). The blood flow is modeled as turbulent, so the Navier-Stokes equation with turbulent terms is utilized [19]:

(2) $$\begin{array}{c} \frac{D{\bar{u}}_{i}}{Dt}=-\frac{1}{\rho }\frac{\partial \bar{P}}{\partial x_{i}}+\frac{\partial }{\partial x_{j}}\left(\frac{\mu +\mu_{T}}{\rho }\left(\frac{\partial {\bar{u}}_{i}}{\partial x_{j}}+\frac{\partial {\bar{u}}_{j}}{\partial x_{i}}\right)\right), \end{array}$$

where *μ* and *μ*_*T*_ are blood viscosity and turbulent viscosity, respectively. The *μ*_*T*_ value depends on the turbulent flow modeling and formulation and is obtained as follows for the *k*-*ω* turbulence model [20]:

(3) $$\begin{array}{c} \mu_{T}=\rho \alpha \frac{k}{\omega }, \end{array}$$

where *k* and *ω* are turbulence kinetic energy and specific turbulence dissipation rates. The following equations [21] must be completely solved to obtain *k* and *ω*.

(4) $$\begin{array}{c} \frac{\partial \left(y^{a}\rho k\right)}{\partial t}+\nabla •\left[y^{a}\left(\rho vk-q_{k}\right)\right]=y^{a}G_{k}, \end{array}$$

(5) $$\begin{array}{c} \frac{\partial \left(y^{a}\rho \omega \right)}{\partial t}+\nabla •\left[y^{a}\left(\rho v\omega -q_{\omega }\right)\right]=y^{a}G_{\omega }, \end{array}$$

(6) $$\begin{array}{c} q_{\omega }=\left(\mu_{0}+\frac{\mu_{T}}{\sigma_{\omega }}\right)\nabla \omega , \end{array}$$

(7) $$\begin{array}{c} q_{k}=\left(\mu_{0}+\frac{\mu_{T}}{\sigma_{k}}\right)\nabla k, \end{array}$$

(8) $$\begin{array}{c} G_{\omega }=\frac{\omega }{k}\left(2\alpha_{\omega }\mu_{T}D^{2}-\beta_{\omega }\rho k\omega +\beta_{\theta }B\right), \end{array}$$

(9) $$\begin{array}{c} G_{k}=2\mu_{T}D^{2}-\beta_{K}\rho k\omega +B, \end{array}$$

(10) $$\begin{array}{c} B=\left(\mu_{0}+\frac{\mu_{t}}{\sigma_{\theta }}\right)\beta g•\nabla \theta , \end{array}$$

(11) $$\begin{array}{c} D=\sqrt{e_{ij}e_{ij}}, \end{array}$$

(12) $$\begin{array}{c} \beta =\frac{-\left(d\rho /d\theta \right)}{\rho }, \end{array}$$

where *D* is the rate of deformation, *β* denotes the coefficient of thermal expansion, *g* is gravitational acceleration, and *θ* denotes the temperature (K). The empirical constants of *α*, *α*_*ω*_, *β*_*K*_, *β*_*ω*_, *σ*_*ω*_, *σ*_*θ*_, *σ*_*ε*_, and *β*_*θ*_ are obtained from Table 1.

The article "Investigation of Artery Wall Elasticity Effect on the Prediction of Atherosclerosis by Hemodynamic Factors" was published in 2022. Journal: Appl Bionics Biomech.

Note that the turbulence intensity (*i*) and the turbulence length scale (*l*) are as follows:

(13) $$\begin{array}{c} i=0.16{\left(\frac{\rho U_{0}D}{\mu }\right)}^{-1/8}, \end{array}$$

(14) $$\begin{array}{c} l=0.07L=0.07D, \end{array}$$

where *D* is vessel diameter, U_0_ is the mean fluid velocity, and *μ* and *ρ* are fluid viscosity and density, respectively. Lagrangian coordinates are used to predict the artery wall displacement. In general, the elastodynamics momentum equation in solids is expressed as follows [23]:

(15) $$\begin{array}{c} \rho_{s}{\ddot{u}}_{s}=\nabla_{0}.\sigma_{s}+\rho_{s}f, \end{array}$$

where *u*_*s*_ is the solid displacement vector, *σ*_*s*_ is the Cauchy stress tensor, *f* is the force vector, and *ρ*_*s*_ is the solid density. Also, in this equation, the gradient is defined based on the moving coordinates and differs from the gradient defined in the fluid mechanics. If the solid is elastic and isotropic and follows Hook's law, the Cauchy stress tensor is expressed as follows:

(16) $$\begin{array}{c} \sigma_{s}=C∶\varepsilon , \end{array}$$

where *C* refers to the quadratic elastic tensor, ∶is a double multiplication sign, and *ε* denote the strain tensor for infinitesimal deformations. But this strain expression method is not suitable for large deformations. Green-Lagrange strain should be used for this purpose. The stress tensor corresponding to this strain is the second-order stress tensor of Piola-Kirchhoff.

(17) $$\begin{array}{c} \sigma_{s}=\frac{1}{J}F.S.F^{T}, \end{array}$$

where *J* is the Jacobian and *F* is the deformation gradient tensor. This tensor involves rotation and deformation. Thus, the Green-Lagrange strain tensor is expressed as follows:

(18) $$\begin{array}{c} E=\frac{1}{2}\left(F^{T}F-1\right). \end{array}$$

At fluid-solid boundary, the fluid–structure interaction (FSI) boundary conditions are as follows [24]:

(19) $$\begin{array}{c} \text{displacement }\left(\text{kinematic condition}\right)\text{: }d_{f}=d_{s}, \end{array}$$

(20) $$\begin{array}{c} \text{shear stress }\left(\text{dynamic condition}\right)\text{: }n\cdot \sigma_{f}=n\cdot \sigma_{s}, \end{array}$$

(21) $$\begin{array}{c} \text{non}–\text{slip condition}:{\dot{d}}_{f}={\dot{d}}_{s}, \end{array}$$

where *d*_*f*_ and *d*_*s*_ are the fluid and solid displacement vectors, respectively, and *σ*_*f*_ and *σ*_*s*_ are the fluid and solid stress tensors, respectively. *n* is the normal vector. For rigid wall, the displacement value is equal to zero. The physical meaning of the above equations is that at the interaction boundary between blood and artery wall, the displacement, normal force, and velocity are equal.

## 4. Boundary Conditions and Numerical Techniques

The displacement and tension of the wall were considered as large in the software and in a solid model for kinematic formulation. The axial and radial motions were fixed at the two ends of the fluid mode and solid. Also, a zero normal stress was applied to the outer artery wall as the boundary condition. In other words, the around tissues applied no external force or pressure to the artery wall [25]. The present work uses the right-side coronary artery pulse flow proposed by Zeng et al. [26], as shown in Figure 2. It had a mean flow rate and a heart period of 1.65 ml/s and 0.8 s, respectively.

The article "Investigation of Artery Wall Elasticity Effect on the Prediction of Atherosclerosis by Hemodynamic Factors" was published in 2022. Journal: Appl Bionics Biomech.

Newton's repetition method was used for both the fluid and the wall models. Furthermore, the sparse solver was utilized to solve the equations. The sparse solver is the advanced version of the Gaussian elimination. It is different from the Gaussian elimination in building solution matrixes. Also, the dispersion of its matrixes is smaller. Actually, it includes only nonzero entries. Consequently, solving equations for zero entries is eliminated, improving the problem-solving rate and reducing the runtime and memory usage for solving the problem [27]. For an elastic wall, the pressure pulse was applied as the boundary condition to the fluid outlet. The same as the velocity pulse, the pressure pulse was obtained from experimental conditions [28].

In the present work, 4 complete cardiac cycles have been used to achieve a steady oscillation solution. Because the results of the third and fourth cycles were similar, the results of the fourth cycle were used [29]. Mechanical deformations in the present study are not large, because studies have shown that the maximum displacement is less than 10% of the original artery dimensions. Hence, the linear elastic assumption is appropriate for the artery wall [30, 31]. Based on the previous studies [9, 17], time steps of 0.001 s, 0.005 s, and 0.01 s were used. Given that the results of time steps of 0.01 and 0.005 (s) were similar, the time step of 0.01 s was selected.

## 5. Model Validation

The present numerical work is a continuation of the experimental work performed by Jahangiri et al. [9, 10]. Jahangiri et al. reported a mismatch between the experimental results and numerical ones (considering laminar flow) for 80% stenosis [9, 10]. Therefore, to increase the accuracy, they used the *k*-*ε* turbulence model. In the present work, the *k*-*ω* turbulence model is used to improve the results of Jahangiri et al. [9, 10]. As shown in Figure 3(a), a great improvement was achieved, especially in specifying the length of reverse flow region.

The solving method should be validated to ensure the numerical solution. It should be noted that the difference between a rigid wall and an elastic wall is in their boundary conditions. Therefore, if the solution is accurate enough for the elastic wall, it can also be used for the rigid wall. Hence, the elastic wall model is used for validation.  Figure 4 compares the numerical and experimental results [32].

The article "Investigation of Artery Wall Elasticity Effect on the Prediction of Atherosclerosis by Hemodynamic Factors" was published in 2022. Journal: Appl Bionics Biomech.

The results of the present study indicate a very good agreement with the experimental ones, especially in the region with the reverse flow (which is the origin of atherosclerosis). Note that that the use of the *k*-*ω* turbulence model in the elastic artery has not been implemented. One of the reasons attributed to the convergence problems occurs in FSI approaches. Because the velocity field was suitably estimated, other hemodynamic parameters can be claimed to be suitably estimated.

To ensure the grid independence of the results, the axial velocity profile was solved for a distance of 1D from the stenosis throat for three grids with different numbers of meshes.  Figure 5 gives the results. As can be seen, the results of a grid with 10200 cells do not significantly differ from those of the cell with 15300 cells. Hence, the computation proceeded with 10200 cells.

As mentioned, blood was considered as a Newtonian fluid. Jahangiri et al. [33] numerically indicated that the error arising from a Newtonian fluid assumption was about 0.6%. Therefore, the Newtonian fluid results can be used with high accuracy.

## 6. Results

Regarding the rigid/elastic and laminar/turbulent scenarios that have been evaluated in the present article, it should be noted that the main purpose was to find the difference between these scenarios for the artery with simple and double stenosis. For example, it has been reported that blood flow through stenosis is turbulent. However, it is not presented how much error there would be in the numerical simulations if the blood flow was assumed to be laminar. It is also obvious that the artery wall is elastic, but in many studies, the artery wall is considered to be rigid, which causes errors in simulation. Therefore, it is necessary to specify the percentage difference between rigid and elastic formulation for hemodynamic parameters. Finally, based on the difference between reality and the simplified assumption, it is mentioned which assumption will impose higher error in the simulation and will lead to more unrealistic predictions.

Hypertension is a factor that influences the intensity of vascular diseases. This has been proved by experiments. Also, it has been suggested that a turbulent flow with high oscillations in the pressure and velocity may damage the plaque [34] or lead to vulnerable plaque rupture [35] because a change in the pressure in pulse flows produces oscillating axial tensile-compressive stresses in deposited plaques, making rupture more likely [36]. Because the knowledge of blood pressure in double stenosis arteries and turbulent blood flow is currently limited, the pressure was investigated to improve the accuracy of clinical diagnosis and decision-making.

The article "Investigation of Artery Wall Elasticity Effect on the Prediction of Atherosclerosis by Hemodynamic Factors" was published in 2022. Journal: Appl Bionics Biomech.

As can be seen, the difference between the rigid and elastic wall results is significant. The elastic wall predicts a lower pressure drop than the rigid wall, which arises from the opening of the elastic wall. In the rigid wall assumption, the pressure reached zero and even negative values for both simple and double stenosis cases. According to Figure 6, it can be said that the rigidity/elasticity of the artery wall is more important than the turbulence model type.

Comparing the results of single stenosis with the results of double stenosis, it can be found that in double stenosis, considering the existence of more obstacles against the blood flow, the upstream pressure is higher, and the upstream conditions become more critical. Also, according to the results, for both rigid and elastic artery cases, the highest rate of blood pressure drop occurs through the throats. Note that the pressure drop for the first throat is higher than the second one. Based on the calculations, it is found that the pressure drop for the former one is greater than the latter one, by 810 Pa (for solid artery) and 540 Pa (for elastic artery). According to the results, after passing through the first and second stenosis owing to the reduction in blood velocity, the pressure rises. Another important point is attributed to the difference between the results of the rigid and elastic arteries. In simple stenosis, the difference is not significant, while in double stenosis, the difference is considerable. In other words, for the case of double stenosis, it is recommended to use the elastic artery formulation.

Figures 7 and Figure 8 show velocity profiles at the time of maximum velocity (3.25 s) for simple stenosis and double stenosis, respectively.

As can be seen, the rigid wall predicts larger maximum velocities than the elastic wall at all locations, but both walls estimate the same reverse flow zone length. It should be noted that the rigid wall shows a slightly larger maximum negative velocity than the elastic wall.

The importance of blood flow velocity consideration is due to the fact that velocity profile has a decisive role in the amount of shear stress on the artery wall. Also, reverse flow regions, which are characterized by a negative velocity value, play a decisive role in the progress of atherosclerosis disease [37–40]. The most important point in Figures 7 and 8 is the maximum velocity of the blood flow through the throats owing to the narrowing in these zones. The maximum velocity is much higher than 1(m/s) (which is the normal biological blood velocity) and therefore can disrupt the circulatory system [41]. Regarding double stenosis, based on the velocity profiles, it is affirmed that the zone between the former stenosis and the latter one is affected by the reverse flow, which can create new stenosis in this zone. In addition, due to the reverse flow between the two stenosis, the maximum velocity in the latter stenosis is higher than the former one.

The article "Investigation of Artery Wall Elasticity Effect on the Prediction of Atherosclerosis by Hemodynamic Factors" was published in 2022. Journal: Appl Bionics Biomech.

In a cardiac cycle, endothelial cells are permanently subjected to different shear stresses. These cyclic changes are defined as OSI [42–43]. The stenosis risk is directly dependent on OSI [45]. It has been suggested that OSI can suitably predict disease risk, compared to clinical data. The results revealed that for simple stenosis, the length of the diseases prone zone in the elastic artery formulation is 21% longer than the rigid one. This figure for double stenosis is calculated to be about 40%.

The research has shown that the high oscillating WSS causes fatigue waste in the intima layer, atherosclerosis, and artery stenosis [46, 47]. Also, mean WSS is a widely used and suitable criterion for flows. It is used to evaluate the total WSS in a cardiac period [48].  Figure 9 demonstrates the effect of artery wall rigidity/elasticity on OSI and mean WSS.

As can be seen in OSI diagrams, the rigid and elastic walls show almost the same reverse flow zone length, but the elastic wall shows larger disease-prone regions as it has a larger OSI > 0 zone. It has been suggested that high OSI regions have distributed endothelial and atherogenesis performance [46, 49].

Furthermore, according to the mean WSS diagrams, the rigid wall shows a larger maximum WSS value, but it does not differ from the elastic wall in other aspects such as the reverse flow zone length. Although a mean WSS of below 0.4 Pa has been known as a factor for endothelial phenotype extension [50], it has been suggested that a mean WSS of above 40 Pa directly damages the endothelial and enhances thrombosis risk [51]. According to the results, both endothelial phenotype extension and thrombosis risk enhancement are observed in the rigid and elastic wall cases. However, the thrombosis risk is higher in the rigid wall assumption.

It is clear that for double stenosis, the difference between the results of the rigid and elastic artery formulation is greater than the case of simple stenosis so that this difference percent can be up to 2.5 times. The maximum amount of mean WSS in the case of simple stenosis (approximately 70 Pa) is higher than double stenosis (approximately 60 Pa) which implies that in simple stenosis the probability of the damage to the endothelial cells and thrombosis is higher than the case of double stenosis. For the case of double stenosis, the maximum mean WSS occurs on the first throat. Also, the area between the two stenosis has a negative mean WSS, which is in agreement with of the velocity profile results.

The article "Investigation of Artery Wall Elasticity Effect on the Prediction of Atherosclerosis by Hemodynamic Factors" was published in 2022. Journal: Appl Bionics Biomech.

The circumferential stress is the stress applied by the fluid to the circumference of the artery. It is important to investigate the circumferential stress because some studies mentioned the role of the increased circumferential stress in the production of the TGF-*β* growth factor by endothelial cells and smooth muscle cells [52]. The increased TGF-*β* growth factor can influence the proliferation of smooth muscle cells, increase smooth muscle cell production enhancement, and extracellular matrix production enhancement. With the enhancement of circumferential stresses in the prestenotic zone (in both simple and double stenosis), one can predict that the wall thickness will increase. This was observed in previous works [52].  Figure 10 compares the circumferential stresses of the rigid and elastic walls. These results were obtained in the last period.

The results suggest that the circumferential stress was larger in the elastic wall than in the rigid wall. This was consistent with previous works [9, 10].  Figure 11 compares the circumferential stress of the rigid and elastic walls in double stenosis.

According to the results, the least circumferential stress on the elastic artery wall occurs at throats, which is attributed to the thicker artery wall and lower displacement at this point. This implies that the lowest production of smooth muscle cells occurs at the throats. In the poststenosis region, circumferential stress increases again, and the thickness of the artery wall rises, with a lower rate than the throat upstream. Comparing the results of the simple stenosis with double, one affirmed that the artery wall thickness growth for the case of double stenosis is greater than that of the single one.

The most probable fluid mechanics parameter related to the beginning and development of vascular diseases is shear stress [53, 54]. The shear stress applied to endothelial cells influences the plaque formation location [55]. A high WSS is known as an important destabilizer acting through variations induced in endothelium and plaque matrix smooth muscle cells [56]. Clinical evidence suggests that WSS not only influences the initial mechanism of plaque appearance [57, 58] but also plays an important role in its development [56]. Endothelial cells subjected to a large WSS take the flow direction, while those subjected to a low or oscillating WSS mostly become round and not in the flow direction. In these regions, cell permeability rises, increasing plaque vulnerability [59]. Considering the abovementioned, it is more important to investigate WSS. Therefore, to observe the importance of the rigid/elastic wall assumption, shear stress is drawn and evaluated for different locations in simple and double stenosis.  Figure 12 compares the WSS of the rigid and elastic walls in simple stenosis. It should be noted that the shear stress values were obtained in the last second. Also, Figure 13 compares the WSS of the rigid and elastic walls in double stenosis.

The article "Investigation of Artery Wall Elasticity Effect on the Prediction of Atherosclerosis by Hemodynamic Factors" was published in 2022. Journal: Appl Bionics Biomech.

As can be seen, the results of the rigid and elastic walls become closer in locations that are far from the reverse flow zone. Therefore, it can be concluded that it is important to assume an elastic wall for modeling zones with reverse flows. It can also be said that the difference between the shear stresses in rigid and elastic walls is smaller in simple stenosis than that in double stenosis.

Concerning WSS, it should be noted that not only a large WSS but also a small WSS is important. It was suggested that a small WSS leads to the residence, adhesion, and infiltration of macromolecules or blood cells to the artery wall [57]. Low WSS regions not only undergo the adhesion of monocytes to endothelium but also lead to endothelial apoptosis in the initial stages of atherogenesis [46, 50, 60] and even stimulate MCP-1 and PDGF-A expressions [61], which leads to the development of atherosclerosis [62]. It was also suggested that when WSS is below 0.4 Pa [50], atherogenic phenotypes, which are related to high OSI in arteries, are stimulated [63, 64].

## 7. Considerations and Limitations

The limitations of the ADINA software are as follows:

- The blood flow through the stenosis is usually turbulent and non-Newtonian. In the ADINA software, for the turbulent regime, there is only the Newtonian option
- The blood flow is laminar before the stenosis throat, and it becomes turbulent by passing through it. In this software, it is not possible to use laminar flow equations for the prestenosis region and turbulent flow equations after the stenosis region
- To satisfy the continuity equation, the displacement of the inlet and outlet of the artery is considered to be zero. This means that to check the parameters, the results should be examined in places that are far enough from the input and output to minimize the effects of input and output
- Also, the plaques considered in the present work are stable. The unstable plaques, which have a lipid core and a fibrous coating with different properties from the artery wall, are very difficult to simulate

The article "Investigation of Artery Wall Elasticity Effect on the Prediction of Atherosclerosis by Hemodynamic Factors" was published in 2022. Journal: Appl Bionics Biomech.

## 8. Conclusion

Vascular diseases are one of the most important causes of death in today's world. Therefore, it is of great importance to identify the factors that cause and develop these diseases. Atherosclerosis is one of the most common arterial diseases, in which fat aggregates in some locations on the artery wall and reduces the cross-section, leading to stenosis. Stenosis changes the motion of blood, which can intensify the disease. Stenosis causes and locations can be detected through parameters such as pressure, effective wall shear stress (WSS), and oscillatory shear index (OSI). The present study numerically investigated turbulent pulse blood flows inside rigid- and elastic-walled arteries with simple and double stenosis. Experimental physiological pulses were used as inlet and outlet boundary conditions. Also, the turbulence *k*-*ω* model was used to obtain hemodynamic parameters. Comparing rigid and elastic wall results indicated as follows:

- The elastic wall predicted a much larger pressure drop that the rigid wall did
- According to the velocity diagrams for simple and double stenosis, the rigid wall predicted a larger maximum velocity than the elastic wall, but both walls gave the same reverse flow zone length
- According to the OSI diagrams, the rigid and elastic walls showed almost the same reverse flow zone length, but the elastic wall showed larger disease-prone locations as it had a larger OSI > 0 zone. Also, according to the mean-time WSS diagrams, the rigid wall showed a larger maximum shear stress. The rigid and elastic wall showed no difference in other aspects, such as the reverse flow zone length
- According to the circumferential stress diagrams of the rigid and elastic walls, the circumferential stress reached its minimum value in the throat and remained almost unchanged after the throat. The results suggested that the circumferential stress was larger in the elastic artery than in the rigid artery

Based on the results, it can be concluded that the turbulence model type has a larger influence than the rigidity or elasticity of the artery. However, this is not the case in some cases, such as axial pressure drop.

## Figures and Tables

**Figure 1:** Calculation domain for an artery with (a) simple stenosis and (b) double stenosis.

**Figure 2:** Mean incoming velocity profile.

**Figure 3:** Pressure pulse applied at outlet boundary [28].

**Figure 4:** Velocity profile at a distance of (a) 1D from the stenosis throat, (b) 1.5D from the stenosis throat, and (c) 2.5D from the stenosis throat.

The article "Investigation of Artery Wall Elasticity Effect on the Prediction of Atherosclerosis by Hemodynamic Factors" was published in 2022. Journal: Appl Bionics Biomech.

**Figure 5:** Grid independency of the results.

**Figure 6:** The axial pressure drops of the rigid and elastic walls.

**Figure 7:** Comparing the velocity profile between the rigid and elastic walls for simple stenosis.

**Figure 8:** Comparing the velocity profile between the rigid and elastic walls for double stenosis.

**Figure 9:** Comparing hemodynamic parameters between the rigid and elastic walls for simple and double stenosis.

**Figure 10:** Comparing the circumferential stresses of the rigid and elastic walls in simple stenosis.

**Figure 11:** Comparing the circumferential stresses of the rigid and elastic walls in double stenosis.

**Figure 12:** Comparing the WSS of the rigid and elastic walls in simple stenosis.

**Figure 13:** Comparing the WSS of the rigid and elastic walls in double stenosis.

**Table 1:** Empirical constants [22].

*α* = 1	*α*_*ω*_ = 0.555	*β*_*k*_ = 0.09	*β*_*ω*_ = 0.075
*σ*_*ω*_ = 2	*β*_*θ*_ = 0.712	*σ*_*θ*_ = 1	*σ*_*k*_ = 2

## Data Availability

All data used to support the findings of this study are included within the article.

## Nomenclature

*g*: Gravitational acceleration (m/s^2^)
*P*: Fluid (blood) pressure (Pa)
*V*: Blood velocity vector (m/s)
*U*_0_: Mean fluid velocity (m/s)
*L*_st_: Length of stenosis region (m)
*R*(*z*): Radius of artery in the stenosis region (m)
*R*_0_: Radius of the healthy artery (m)
*R*_0,*t*_: Radius of artery at the stenosis throat (m)
*z*: Axis coordinates of stenosis (m)
*z*_*m*_: Axis coordinates of stenosis throat from the origin of coordinates (m)
*t*: Time (s)
*β*: Coefficient of thermal expansion
*θ*: Temperature (K)
*F*: Deformation gradient tensor (-)
*E*: Green-Lagrange strain tensor (-)
*d*_*s*_: Solid displacement vector (m)
*d*_*f*_: Fluid displacement vector (m)
*σ*_*s*_: Solid stress tensor (N/m^2^)
*σ*_*f*_: Fluid stress tensor (N/m^2^)
*i*: Turbulence intensity
*l*: Turbulence length scale (m)
*D*: Artery diameter (m)
*L*: Length of artery (m)
*ρ*: Density (kg/m^3^)
*μ*_*T*_: Turbulence viscosity (Pa.s)
*μ*: Blood viscosity (Pa.s)
*K*: Turbulence kinetic energy (m^2^/s^2^)
*ϵ*, *ω*: Specific turbulence dissipation (m^2^/s^3^)
OSI: Oscillatory shear index
WSS: Mean shear stress (Pa).
